# Dynamic Monitoring of Serum Protein in Acute Respiratory Distress Syndrome Based on Artificial Neural Network

**DOI:** 10.1155/2022/3542942

**Published:** 2022-10-17

**Authors:** Zhihui Zhou, Yi Long

**Affiliations:** ^1^Department of Critical Care Medicine, Chongqing General Hospital, Chongqing 401120, China; ^2^Department of Critical Care Medicine, Chongqing University Cancer Hospital, Chongqing 400030, China

## Abstract

Acute respiratory distress syndrome (ARDS) is one of the more serious diseases in human lung disease. Reducing its incidence rate is an important task in current clinical research. Dynamic monitoring of serum protein in patients will help to achieve the early diagnosis and treatment of ARDS. In this study, a protein monitoring model based on artificial neural network is proposed. First, surface enhanced laser desorption ionization time-of-flight mass spectrometry is used for protein detection, and then BP neural network is used for protein classification and content analysis. In the experimental analysis, serum samples from patients with acute respiratory distress syndrome in our hospital from November 2020 to August 2021 were selected for experimental testing. The experimental results show that the serum protein monitoring model based on BP neural network has low error and high convergence ability and can monitor individual protein in protein monitoring, and the area under the ROC curve in diagnostic performance reaches 0.854. The above results show that the artificial neural network has a good effect on the dynamic monitoring of serum protein in acute respiratory distress syndrome, and the diagnostic performance evaluation can reach 0.854, which has the ability to significantly improve the clinical diagnosis and treatment of acute respiratory distress syndrome.

## 1. Introduction

Acute respiratory distress syndrome (ARDS) is an acute inflammation of the lungs. The mortality of patients with severe ARDS can be as high as 50%. After years of clinical research and practice, the known causes of severe acute respiratory distress syndrome are complex and diverse. In clinical practice, severe infection and trauma are the main causes of the disease. Therefore, acute respiratory distress syndrome is the main factor causing respiratory failure [1–3]. Acute respiratory distress syndrome will show rapid deterioration at the initial stage of onset, and its deterioration will cause severe damage to patients. Therefore, it is an important research content to target acute respiratory distress syndrome in clinical practice [4, 5]. It is of great significance to treat and block respiratory distress syndrome at the stage of disease development. At present, acute physiology and chronic health scoring tools are generally used for clinical diagnosis of respiratory distress syndrome. However, the complexity of clinical diagnosis and the impact of subjective operation make it difficult to meet clinical needs [6–8]. On this basis, with the continuous development of medical technology, for patients with acute respiratory distress syndrome, serum protein detection has gradually become the main means of clinical diagnosis of acute respiratory distress syndrome [9].

In recent years, with the increasing incidence rate of acute respiratory distress syndrome, improving the clinical diagnostic effect of acute respiratory distress syndrome has become an important means to alleviate the disease. Among them, serum protein monitoring through proteomics technology is a more effective method [10, 11]. Clinical proteomics technology is a medical technology to study the changes of human protein. In clinical proteomics technology, surface enhanced laser desorption ionization technology can directly detect blood, urine, and other samples [12, 13]. In protein detection, surface enhanced laser analytic ionization can analyze the dynamic changes of disease-specific proteins, show the content of proteins in the test samples and the molecular weight information, and compare the protein differences between the disease samples and the normal samples, so as to obtain the early disease indicators and symptoms [14, 15]. In order to improve the clinical diagnostic effect of acute respiratory distress syndrome, most studies have proposed a serum protein monitoring scheme for patients with acute respiratory distress syndrome. However, from the current application status, in the information age, a large number of serum protein monitoring methods are slightly backward. How to realize intelligent monitoring is a problem that needs to be solved in clinic [16].

With the continuous development of the information age, intelligent medicine has gradually attracted people's attention, and artificial intelligence technology has also been widely used in medical diagnosis and treatment. In the application of artificial intelligence technology, deep learning is particularly widely used because it can continuously improve the self-detection performance by using the adaptive learning ability in disease diagnosis and greatly improve the disease diagnosis ability in intelligent medicine [17–19]. In medical diagnosis and treatment, as an advanced computer network algorithm, artificial neural network (ANN) can effectively analyze complex data by simulating biological intelligent processing ability [20]. At the same time, in the process of in-depth learning, the use of artificial intelligence algorithms to achieve human physiological indicators has gradually become an important technology in the current intelligent medicine [21]. However, the application and effect of most artificial intelligence algorithms in intelligent medical treatment are still difficult to meet the needs of medical treatment. Therefore, the application of artificial neural network in medical diagnosis is deeply discussed in this research.

In the diagnosis of acute respiratory distress syndrome, artificial neural network technology will be used to realize the dynamic monitoring of serum protein. In order to monitor the acute respiratory distress syndrome accurately and dynamically, BP neural network of artificial neural network was used to realize the dynamic monitoring of serum protein. BP neural network uses direction propagation to process information. In the process of direction propagation, BP neural network can minimize the error between the actual output and the expected value. Therefore, in this study, the dynamic monitoring of serum protein was carried out by surface enhanced laser desorption ionization, and the diagnostic model of acute respiratory distress syndrome was established by using the low error ability of BP audit network.

## 2. Related Work

### 2.1. Acute Respiratory Distress Syndrome Protein Monitoring

Due to the serious consequences of acute respiratory distress syndrome, in order to understand its pathogenesis, a large number of studies have given monitoring results for the protein changes in the course of its pathogenesis. Cui et al. analyzed the influence mechanism of death-related protein kinase 1 in acute respiratory distress syndrome, monitored the change of death related protein kinase 1 under 5-Aza-2′- deoxycytidine, and evaluated the effect of related protein change on acute respiratory distress syndrome [22]. Ortolan et al. found through research that the change of endothelial protein C receptor is an important risk factor in the pathogenesis of acute respiratory distress syndrome. Using protein monitoring technology, they learned that the change of endothelial protein C receptor will increase cell adhesion, and the improvement of cell adhesion is the main influencing factor of acute respiratory distress syndrome [23]. In order to understand the pathogenesis of acute respiratory distress syndrome, Dahmer et al. found that the increase of surfactant protein D is a relatively specific indicator of lung injury through protein monitoring and proved that the increase of surfactant protein D is related to the poor prognosis of children with acute respiratory failure through the design of relevant experiments [24]. Svenja et al. developed Luminex binding analysis to realize high-throughput and rapid serum protein monitoring in patients with acute respiratory distress syndrome and rapidly detected circulating antibodies to coronavirus type 2 s protein in patients with acute respiratory distress syndrome, which facilitated the prognosis of acute respiratory distress syndrome [25].

In the early diagnosis of acute respiratory distress syndrome, dynamic monitoring of protein can effectively predict the onset of acute respiratory distress syndrome. However, it can be found from the existing studies that few studies can monitor multiple proteins at one time in the dynamic monitoring of proteins, and the monitoring results of existing studies are difficult to meet the clinical needs.

### 2.2. BP Neural Network

As a traditional artificial neural network, BP neural network has a good computing ability and classification ability. With the development of society, its application field is gradually expanding. In order to improve the effect of information processing and reduce the loan and storage resources of information in the transmission process, Yang et al. proposed an image compression and encryption algorithm based on BP neural network, which uses the information processing technology of BP neural network to compress the information and increase the security of information in transmission [26]. Ghosh et al. used the artificial neural network to diagnose cardiovascular diseases, estimated the characteristics of cardiac health monitoring parameters for patients, realized the screening of cardiac disease precursors, and combined the artificial neural network with impedance cardiogram to check individual cardiovascular health [27]. Li et al. proposed a small sample learning method based on data expansion and a GA based method for fault diagnosis of high pressure common rail diesel engine. The fault diagnosis method of BP neural network uses the data processing ability of neural network for fault diagnosis. The results show that the overall accuracy of the fault diagnosis model based on the improved BP neural network is as high as 98.3% [28]. In order to realize the intelligent classification of loess deposits in tunnel engineering, Zhang and others proposed an evaluation system based on BP neural network, which was applied to practical analysis and showed that the model output results were consistent with the actual results [29].

Artificial neural network has been gradually applied in many fields, but it is rarely used in medical assistance. Therefore, BP neural network of artificial neural network is applied to the dynamic monitoring of protein in acute respiratory distress syndrome in order to improve the early diagnosis effect of acute respiratory distress syndrome.

## 3. Method

### 3.1. Dynamic Monitoring Technique of Surface Enhanced Laser Analytical Ionization

Surface enhanced laser desorption ionization is a rising technology in the development of proteomics. It is often combined with time-flight mass spectrometry in application and has a good dynamic detection effect on specific proteins in serum samples. The whole technical process of surface enhanced laser desorption ionization time-flight mass spectrometry is shown in Figure 1.

As shown in Figure 1, surface enhanced laser desorption ionization time-of-flight mass spectrometry is a combination of chip technology and mass spectrometry technology. Its technical process includes selecting protein chip carrier, selecting and fixing probe, preprocessing of serum samples, chip detection, and computer data processing [30]. Surface enhanced laser desorption ionization time-of-flight mass spectrometry has the characteristics of strong specificity and high resolution in protein detection and can detect low abundance and small molecular weight proteins, as well as disease-related protein changes.

In the diagnosis and treatment of lung diseases, surface enhanced laser desorption ionization time-of-flight mass spectrometry has been gradually applied to the classification and prediction of lung cancer tissues and the diagnosis of lung cancer. Some studies have confirmed that surface enhanced laser desorption ionization time-of-flight mass spectrometry can effectively detect the malignant protein signal of lung epithelial cells and has important value in the diagnosis and screening of lung cancer [31, 32]. However, the application of surface enhanced laser desorption ionization time-of-flight mass spectrometry still needs to be improved. First, surface enhanced laser desorption ionization time-of-flight mass spectrometry is a semiquantitative technology, and the difference in protein properties and serum concentration shown in the detection cannot be shown [33]. Second, the protein sequence cannot be classified and analyzed, that is, the protein sequence cannot be determined, resulting in the inability to obtain important information such as protein configuration in protein detection [34].

### 3.2. A Diagnosis Model Based on BP Neural Network

After protein detection by surface enhanced laser desorption ionization time-of-flight mass spectrometry, BP neural network model was constructed and trained by using the detection results. Each node of BP neural network represents a specific function, and the connection between the two nodes represents the weight. It is worth noting that BP neural network will continuously adjust the weight during long-term learning to optimize the data processing performance of the model [35, 36]. In order to improve the data processing performance of BP neural network, a three-layer BP neural network model is constructed as shown in Figure 2.

It can be seen from Figure 2 that the number of input neurons and output neurons of the three-layer BP neural network model used in the study is set as *m* and *p* in turn, and the number of hidden layer neurons is *n*. At this time, the *m*-th neuron in the existing input layer is expressed as *x*_*m*_, and the *n*-th neuron in the hidden layer and the *p*-th neuron in the output layer are expressed as *z*_*n*_ and *y*_*p*_ in turn. *W*_*mn*_ represents the connection weight from the input layer to the hidden layer, and *W*_*np*_ represents the connection weight from the hidden layer to the output layer. The selection of hidden layer neurons is shown in the following formula.

(1) $$\begin{array}{c} n<\sqrt{m+p}+a. \end{array}$$

Equation (1) is the empirical formula for selecting the reference of the number of neurons in the hidden layer *n*, where *m* represents the number of nodes in the input layer, *p* represents the number of nodes in the output layer, and *a* represents any constant in the interval (0, 10). Second, sigmoid function in BP neural network is analyzed, as shown in the following formula.

(2) $$\begin{array}{c} f\left(x\right)=\frac{1}{\left(1+e^{-x}\right)}. \end{array}$$

Equation (2) is the sigmoid type nonlinear function *f*(*x*) acting on each neuron, and *x* is the input function value. Through the hidden layer, the output of BP neural network is obtained, as shown in the following formula.

(3) $$\begin{array}{c} \left\{\begin{array}{c} {\text{net}}_{k}=\underset{j}{\sum }\omega_{kj}O_{j}+\theta_{k},\\ O_{k}=f\left({\text{net}}_{k}\right). \end{array}\right. \end{array}$$

In formula (3), *ω*_*kj*_ represents the connection weight value between neuron *U*_*k*_ and upper layer neuron *U*_*j*_; *O*_*j*_ represents the output of neuron *U*_*j*_. The input value, output value, and threshold value of neuron *U*_*k*_ are represented by net_*k*_, *O*_*k*_, and *θ*_*k*_ in turn. When BP neural network is used as a weak learning model, and the loss function is *ψ*(*y*, *f*) = 1/2 · (*y* − *f*(*x*))^2^ at the same time, the residual error is (*y* − *f*(*x*)), where *f*(*x*) is the model fitting value. Continue to fit the residuals, and train the next BP neural network along the descending direction of the gradient.

(4) $$\begin{array}{c} \hat{f}\left(x\right)=f_{0}\left(x\right)+\overset{M}{\underset{i=1}{\sum }}\rho_{i}\cdot h\left(x,\theta_{i}\right). \end{array}$$

Equation (4) is the calculation formula of the model fitting value of the test data, where *ρ*_*i*_ represents the optimal reduction step, *h*(*x*, *θ*_*i*_) represents the weak learning model, *θ* represents the model parameters, and *M* represents the number of iterations.

### 3.3. Experimental Design

All data in the study are from November 2020 to August 2021, and all samples are from inpatients in our hospital. Inclusion criteria: (1) meet the diagnostic criteria of acute respiratory distress syndrome; (2) complete clinical data. Exclusion criteria: (1) patients with chronic obstructive pulmonary disease; (2) liver and kidney dysfunction; (3) used glucocorticoids.

Collect 3 ml of fasting venous blood of the subjects, store the serum samples in a 4°C refrigerator, and centrifuge the serum samples for 5 min after standing for 1 h. The centrifuged serum was centrifuged again for 5 min, and the serum was subpacked and stored in a -80°C refrigerator. At the same time, the sera of normal people were collected and mixed. They were used as the mixed control group and stored in the refrigerator at -80°C.

The serum samples were detected by surface enhanced laser desorption ionization time-of-flight mass spectrometry chip. The serum protein mass spectra of acute respiratory distress syndrome and normal control group were detected, respectively. The serum protein on the surface of the serum protein chip was detected. The mass charge ratio range of the chip was optimized to be 2000~20000 m/z, and the laser intensity was 210. Baseline reduction and homogenization were used to preprocess the obtained serum protein mass spectra. The BP neural network is used to build the diagnosis model. In the diagnosis model, the nodes of the input layer, hidden layer, and output layer of the BP neural network model are set as 5, 4, and 1, respectively. The tangent S-shaped transfer function is used in the operation of BP neural network, and the operation results are initialized randomly in the calculation. In the input node, the peak intensity of the screened differential protein is used as the input.

## 4. Results

### 4.1. Repeatability Test Results

The obtained serum protein mass spectrum data are shown in Figure 3. It can be seen from Figure 3 that in order to avoid the interference of matrix peaks on the repeatability test results, the peaks below 2000 m/z are filtered. In the expression of serum protein mass spectrometry data, the protein peaks with strong expression were 2735 m/z, 4080 m/z, 6970 m/z, and 7010 m/z, respectively. The average coefficient of variation of the four peaks was 13.64%, which was below 15%, indicating a high repeatability. At the same time, it can be seen that 2735 m/z appears in each map, and the average coefficient of variation is 14.32%, which is less than 15%.

### 4.2. Detection of Differential Protein Peaks

The sera of patients with acute respiratory distress syndrome and the control group were analyzed by surface enhanced laser desorption ionization time-of-flight mass spectrometry. A total of 794 protein peaks were detected, as shown in Figure 4. As can be seen from Figure 4, in the difference analysis between the two groups, the statistical analysis results showed that there were significant differences in 118 protein peaks between the two groups, and the test results showed that the differences were statistically significant (*p* < 0.05). It can be seen that the peak of serum protein mass charge ratio in patients with acute respiratory distress syndrome and the control group is mainly distributed between 2000~15000 m/z.

It can be seen from Figure 4 that in the comparison of serum differences between patients with acute respiratory distress syndrome and the control group, 15 protein peaks are distributed between 2000 and 8000 m/z. Through statistical analysis, it can be found that in the expression of serum proteins in patients with acute respiratory distress syndrome and the control group, the differences of 15 protein peaks in the classification cluster are particularly obvious. The comparison results are shown in Figure 5.

### 4.3. Performance Analysis of BP Neural Network

The 15 protein peaks with significant differential expression are used for combination processing, and the BP neural network protein monitoring model is constructed. The performance of the constructed protein monitoring model based on BP neural network is analyzed. First, the mean square error (MSE) of BP neural network in the training process is analyzed, as shown in Figure 6. As can be seen from Figure 6, with the increasing number of iterations, the mean square error of BP neural network protein monitoring model shows a decreasing trend. After the number of iterations reaches 20, the curve decreasing speed gradually decreases. After the number of iterations reaches 80, the mean square error of the model approaches the target value and begins to remain stable.

Figure 7 shows the change results of the fitness values of the BP neural network protein monitoring model. From Figure 7, it can be seen that the BP neural network and the convolution neural network are compared and analyzed. With the increase of iteration times, the number of iterations required to reach the optimal fitness of the BP neural network model is significantly less than that of the convolution neural network. The above results show that compared with convolution neural network, BP neural network can reach the best fitness faster in data processing and has better convergence.

### 4.4. Effect Analysis of BP Neural Network Protein Monitoring Model

Select 10 patients with acute respiratory distress syndrome and 10 normal people for BP model monitoring, diagnosis, and test analysis, as shown in Table 1. It can be seen from Table 1 that the BP neural network protein monitoring model can be used to calculate the output value for patients with acute respiratory distress syndrome and the normal population, and the difference between the output value and the target output value is not obvious, indicating that the status of acute respiratory distress syndrome of the tested population can be accurately judged.

BP neural network was used to monitor the protein of the subjects. During the monitoring process, the difference between the serum protein of patients with mild, moderate and moderate acute respiratory distress syndrome, and the normal population was compared, as shown in Table 2. It can be seen from Table 2 that the monitoring includes C-reactive protein (CRP) and albumin (ALB). Table 2 shows that under the BP neural network protein monitoring model, the serum protein content of patients with acute respiratory distress syndrome can be clearly displayed and can be significantly distinguished from the normal population.

Finally, the diagnostic performance of BP neural network protein monitoring model in the diagnosis of acute respiratory distress syndrome is analyzed, as shown in Figure 8. As can be seen from Figure 8, the offline area of BP neural network model is 0.854, significantly larger than 0.5, with good diagnostic performance.

## 5. Discussion

In order to diagnose acute respiratory distress syndrome, according to the changes of physiological characteristics of patients with acute respiratory distress syndrome, artificial neural network was used to monitor the serum protein of patients. In the research, first, the protein of the research object is detected by surface enhanced laser desorption ionization time-of-flight mass spectrometry. Second, the BP neural network model is used to realize protein classification and protein level content analysis. Finally, the effectiveness of the proposed model is obtained through experimental tests.

In the study, aiming at the application effect of surface enhanced laser desorption ionization time-of-flight mass spectrometry, the effectiveness of surface enhanced laser desorption ionization time-of-flight mass spectrometry was analyzed through repeatability test and differential protein peak detection. The results show that in the repeatability test, the average coefficient of variation between multiple chips is 13.64%, which has high repeatability; The detection of differential protein peak shows that there is a significant difference in serum protein expression between patients with acute respiratory distress syndrome and normal people, and the above results are consistent with the results of previous studies [37].

The performance analysis of BP neural network model shows that its error value continues to decrease with the increase of iteration times and can reach the target value after fewer iterations, indicating that it has high convergence and can improve the efficiency of the diagnostic model. The comparative analysis of model fitness shows that compared with convolutional neural network, BP neural network can reach the best fitness faster, indicating that BP neural network has better convergence and higher adaptability. The current research results are consistent with previous studies [38]. The protein monitoring model based on BP neural network model is applied to clinical practice. The results show that the BP neural network protein monitoring model can clearly show the numerical difference between patients with acute respiratory distress syndrome and normal people, that is, it can accurately distinguish the two and achieve the effect of preoperative diagnosis. Analyzing the diagnostic performance of BP neural network protein monitoring model, the ROC curve shows that the area under the curve of BP neural network protein monitoring model is as high as 0.854, indicating that this model has a significant effect in diagnosing acute respiratory distress syndrome by monitoring serum protein content [39].

In conclusion, it is effective to use artificial neural network to monitor the serum protein of patients with acute respiratory distress syndrome, and it can make early diagnosis of acute respiratory distress syndrome. However, there are still some limitations in the study. The proteome in serum is complex and diverse, and the protein types monitored in the study are still few. In the follow-up work, it is necessary to monitor other serum protein types.

## Figures and Tables

**Figure 1:** Technical process of surface enhanced laser desorption ionization time of flight mass spectrometry.

**Figure 2:** Schematic diagram of BP neural network.

**Figure 3:** Detection of protein fingerprints in serum samples.

**Figure 4:** Differential expression of serum protein fingerprints in patients with acute respiratory distress syndrome and control group.

**Figure 5:** Difference in expression intensity of 15 protein peaks.

**Figure 6:** Training results of mean square error of BP neural network.

**Figure 7:** Comparison of fitness of different neural network models.

**Figure 8:** ROC curve of BPNN monitoring model.

**Table 1:** Comparison of model experiment results.

Target number	Acute respiratory distress syndrome		Normal	
	Target output value	BP output value	Target output value	BP output value
0	1	0.935642	0	0.027464
1	1	0.975358	0	0.018971
2	1	0.973150	0	0.038612
3	1	1.054531	0	0.027431
4	1	1.131256	0	0.013472
5	1	0.972101	0	0.039412
6	1	0.892345	0	0.019418
7	1	0.987982	0	-0.015646
8	1	0.948542	0	0.223763
9	1	0.963165	0	0.026429
10	1	1.078321	0	0.013494

**Table 2:** Protein detection of BPNN monitoring model.

Group	Acute respiratory distress syndrome			Normal
	Light	Moderate	Severe	
CRP (mg/L)	86.03 ± 12.97	121.39 ± 25.72	152.92 ± 33.01	6.31 ± 1.21
ALB (g/L)	27.83 ± 1.01	26.91 ± 1.04	24.51 ± 2.03	37.31 ± 1.42
CRP/ALB	3.09 ± 0.43	4.69 ± 1.01	6.72 ± 0.42	0.18 ± 0.03

## Data Availability

The dataset can be accessed upon request.
